The article "Mechanism of Mitophagy and Its Role in Sepsis Induced Organ Dysfunction: A Review" was published in 2021. Journal: Front Cell Dev Biol.

# Mechanism of Mitophagy and Its Role in Sepsis Induced Organ Dysfunction: A Review

**DOI:** 10.3389/fcell.2021.664896

**Published:** 2021-06-07

**Authors:** Cheng-long Zhu, Ren-qi Yao, Lu-xi Li, Peng Li, Jian Xie, Jia-feng Wang, Xiao-ming Deng

**Affiliations:** ^1^Department of Anesthesiology and Intensive Care, Changhai Hospital, The Naval Medical University, Shanghai, China; ^2^Trauma Research Center, Fourth Medical Center of the Chinese PLA General Hospital, Beijing, China; ^3^Department of Burn Surgery, Changhai Hospital, The Naval Medical University, Shanghai, China

**Keywords:** mitophagy, mitochondria, sepsis, autophagy, organ dysfunction

## Abstract

Autophagy, an evolutionarily conserved process, plays an important role in maintaining cellular homeostasis under physiological and pathophysiological conditions. It is widely believed that mitochondria influence the development of disease by regulating cellular metabolism. When challenged by different stimuli, mitochondria may experience morphological disorders and functional abnormalities, leading to a selective form of autophagy—mitophagy, which can clear damaged mitochondria to promote mitochondrial quality control. Sepsis is a complex global problem with multiple organ dysfunction, often accompanied by manifold mitochondrial damage. Recent studies have shown that autophagy can regulate both innate and acquired immune processes to protect against organ dysfunction in sepsis. Sepsis-induced mitochondrial dysfunction may play a pathophysiological role in the initiation and progression of sepsis-induced organ failure. Mitophagy is reported to be beneficial for sepsis by eliminating disabled mitochondria and maintaining homeostasis to protect against organ failure. In this review, we summarize the recent findings and mechanisms of mitophagy and its involvement in septic organ dysfunction as a potential therapeutic target.

## Introduction

All living organisms undergo successive renovation. During human growth and development, cells are continuously remodeled and recycled, as well as intracellular components, which is intended to replace the old component with a new component with better quality. Autophagy, initially described as a non-selective nutrient recycling procedure (Anding and Baehrecke, 2017), is a major intracellular degradation mechanism. Cytoplasmic contents are sequestered into autophagosomes, which fuse with lysosomes to degrade their substances via the action of lysosomal hydrolases (Mizushima and Komatsu, 2011). More recently, selective autophagy specifically recognizes and degrades a particular cargo, either a protein complex, an organelle, or an invading microbe, and cells utilize selective autophagy for a variety of purposes, including remodeling to adapt to changing environment or nutritional conditions and to eliminate damaged organelles (Jin et al., 2013). As the “energy center” of the cell, mitochondria produce ATP and many biosynthetic intermediates and have diverse but interrelated functions, while also promote stress responses such as autophagy and apoptosis (Nunnari and Suomalainen, 2012). Mitochondrial dysfunction has become a key factor in numerous diseases, including neurodegenerative diseases, metabolic diseases, and infections. Selective autophagy of mitochondria (called mitophagy) promotes mitochondrial quality control by inducing the clearance of damaged mitochondria through an autophagic mechanism (Ashrafi and Schwarz, 2013; Cho et al., 2020). Importantly, mitophagy plays a pivotal role in determining cell fate by maintaining cellular and mitochondrial homeostasis in inflammatory diseases (Ma et al., 2020).

Sepsis is defined as organ dysfunction caused by a dysregulated host response to infection (Shankar-Hari et al., 2016). We should focus our treatment in supporting organ function when attempting to eliminate the pathogens and inflammation. In sepsis, the long-recognized role of autophagy as a cellular adaptive mechanism is to attenuate cellular injury and apoptosis, and the maintenance of autophagy in sepsis may be helpful in limiting sepsis-induced organ injury. Recently, the organ-protective role of autophagy in sepsis has attracted widespread attention (Yin et al., 2019). During sepsis, mitochondria dysfunction is induced by the presence of large amounts of inflammatory factors. In particular, a series of studies have clarified an important role of mitophagy in organ dysfunction during sepsis. In addition, mitophagy has also been reported to regulate macrophage activity during sepsis in recent years. Kim et al. (2016) found that mitophagy could be induced to inhibit NLRP3 (NLR family pyrin domain containing 3) activation in macrophages to suppress sepsis; however, Patoli et al. (2020) indicated that inhibition of mitophagy powers macrophage activation and defense against bacterial action during sepsis. In this review, we summarize the detailed mechanisms of mitophagy (Figure 1) in mammalian cells as well as its protective role in septic organ dysfunction as underlying therapeutic targets for sepsis.

**FIGURE 1:** Molecular mechanism of mitophagy. PINK1-Parkin -dependent mitophagy. PINK1 serves as a molecular sensor of mitochondrial health, it detects disruptions and signals to recruit and activate parkin, which can then be amplified by ubiquitinating mitochondrial surface proteins. These ubiquitinated proteins can subsequently be recognized by autophagic receptors that convert mitochondria to autophagosomes for degradation via interacting with LC3 protein directly. TBK1 can phosphorylate autophagic receptors to enhance mitophagy. A PINK1-dependent TUFm phosphoswitch determines conversion from activating to suppressing mitophagy. PINK1-Parkin -independent mitophagy. This process is mediated by mitophagy receptor proteins, such as NIX, FUNDC1, BNIP3, owning the unique ability to interact with processed LC3 independent of ubiquitin.

## Cell Death in Sepsis

In sepsis a massive immune cell death can occur especially in lymphocytes, which can be performed in three ways: apoptosis, necrosis, and autophagy (Hotchkiss et al., 2009; Cheng et al., 2020), which contributes to protracted immunosuppression. Apoptosis is a form of programmed cell death that depends on the activity of cystatin and histone proteases, which is thought to play an important role in sepsis-induced organ dysfunction and immune dysregulation (Hotchkiss et al., 2013; Lelubre and Vincent, 2018). Necrosis is a non-programmed, energy-independent form of cell death that can be triggered by a variety of virulence factors released by pathogens. In turn, necrosis may exacerbate local inflammation through extracellular release of “danger signal molecules” (e.g., HMGB1) (Pinheiro da Silva and Nizet, 2009). The role of autophagy in cell death is controversial. Although a large number of autophagic vesicles have been observed in dying cells from different species of animals, what is not clear is whether this aids cell death or is compensated for cell death (Levine and Yuan, 2005; Hotchkiss et al., 2009). Knockdown of key autophagy genes may promote apoptosis, suggesting that autophagy is a self-limiting survival strategy rather than a primary or irreversible death execution program (Boya et al., 2005; Levine and Yuan, 2005).

Apoptosis is the main mechanism of lymphocyte death in sepsis, and regulation of lymphocyte apoptosis is the key to improving sepsis survival (Hotchkiss and Nicholson, 2006). In addition, if autophagy is inhibited, cells may be more susceptible to apoptosis (Boya et al., 2005; Ravikumar et al., 2006). Numerous studies in animals have highlighted that apoptosis can exacerbate sepsis and that prevention of sepsis-induced apoptosis can improve survival, thus suggesting that regulation of immune apoptosis is critical for improving sepsis survival (Hotchkiss and Nicholson, 2006; Ayala et al., 2008). Atg5, an autophagy protein is cleaved by calpain and induces apoptosis by binding Bcl-xL, an anti-apoptotic transmembrane protein component of mitochondria (Luo and Rubinsztein, 2007; Gordy and He, 2012). It is also known that the anti-apoptotic Bcl2/Bcl-xL complex conjugates with Beclin-1 to inhibit autophagy (Pattingre et al., 2005). This implies the importance of regulating the crosstalk between autophagy and apoptosis. Overexpression of anti-apoptotic proteins may permit the survival of injured cells in sepsis, and autophagy may assist by providing key metabolites (Hotchkiss et al., 2009). Autophagy genes may also be critical for maintaining cellular bioenergetics and survival by limiting cell death to the site of infection and enhancing innate immunity (Levine and Yuan, 2005). In addition, the importance of mitochondrial dysfunction in the pathogenesis of organ damage caused by sepsis has been increasingly recognized (Arulkumaran et al., 2016), and mitophagy may increase in early sepsis to limit the deleterious effects of mitochondrial dysfunction (Lelubre and Vincent, 2018).

## Overview of Mitophagy

Functional mitochondria are critical for multiple intracellular processes as the main source of ATP, maintaining cellular integrity and survival, and play a major role in initiating programmed cell death. Mitochondrial dysfunction is defined as diminished mitochondrial biogenesis, changes in membrane potential, decrease in mitochondrial number and altered activity of oxidative proteins due to the accumulation of ROS (reactive oxygen species) in cells and tissues, which markedly disrupts cellular metabolic homeostasis and results in cell death (Bhatti et al., 2017). When damaged mitochondria emerge, a selective form of autophagy, termed mitophagy, will eliminate them, ensuring the maintenance of a healthy cohort of mitochondria. Several mechanisms have been reported to be involved in achieving functional homeostasis of the morphological integrity of mitochondria (Romanello and Sandri, 2015). Mitophagy has a significant role in mitochondrial quality control and is able to alleviate cell death and diseases (Romanello and Sandri, 2015; Von Stockum et al., 2016).

The most widely studied selective autophagy pathway is mitophagy, a mechanism for the selective degradation of mitochondria, which can be initiated through both PINK1 (PTEN induced putative kinase 1)-PRKN (Parkin RBR E3 ubiquitin protein ligase)-dependent and -independent pathways (Yao et al., 2020). PINK1 and Parkin (also known as PARK2) (Durcan and Fon, 2015), play a key role in maintaining mitochondrial health by identifying damaged mitochondria and degrading them. PINK1 is a serine/threonine kinase located exclusively on depolarized mitochondria, while Parkin is a ubiquitin ligase (E3) that catalyzes the transfer of ubiquitin to mitochondrial substrates (Corti et al., 2011; Narendra et al., 2012; Bose and Beal, 2016). PINK1 acts as a molecular sensor of mitochondrial health, constantly surveying mitochondrial status until it detects damage and signals for the recruitment and activation of Parkin. In healthy mitochondria, the mitochondrial transmembrane potential drives the import of PINK1 into the IMM (inner mitochondrial membrane) via OMM (outer mitochondrial membrane) and IMM translocases (TOMM and TIMM, respectively) (Nguyen et al., 2016). Recently, PINK1 was found to interact with the autophagic effector TUFm (mitochondrial Tu translation elongation factor) and phosphorylate TUFm at Ser222, and the self-antagonistic function of PINK1/TUFm is essential for the homeostasis of mitophagy regulation (Lin et al., 2020). In the cytosol, Parkin remains inactive and adopts an autoinhibited conformation (Trempe et al., 2013). When damage occurs in mitochondria, PINK1 phosphorylates Parkin at S65 in the UBL domain and this has been demonstrated to stimulate the activity of Parkin’s ligase and recruitment to mitochondria (Kondapalli et al., 2012; Shiba-Fukushima et al., 2012).

To ensure efficient mitophagy, many mitophagy receptors (Table 1) are essential, such as OPTN (optineurin) (Heo et al., 2015), SQSTM1/p62 (sequestosome 1) (Yamada et al., 2019), CALCOCO2/NDP52(calcium binding and coiled-coil domain 2) (Goiran et al., 2018), MFN1 (mitofusin 1), MFN2 (mitofusin 2) (Chen and Dorn, 2013; Song et al., 2015) and TAX1BP1 (Tax1 binding protein 1) (Heo et al., 2019). Despite the presence of basal ubiquitin proteins on the OMM, autophagy receptors do not recruit mitochondria in the absence of mitochondrial damage. The intrinsic interaction of TBK1 (TANK binding kinase 1) with OPTN and the ability of OPTN to attach to the ubiquitin chain are critical for TBK1 recruitment and kinase activation to mitochondria. In turn, TBK1 phosphorylates OPTN at S473, thereby extending the binding capacity of OPTN to diverse Ub (ubiquitin) chains (Richter et al., 2016). SQSTM1/p62 is thought to function as an autophagy receptor that connects autophagy substrates and autophagosomes by binding both ubiquitin and MAP1LC3/LC3 (microtubule associated protein 1 light chain 3) (Katsuragi et al., 2015). When cytotoxic proteins aggregate, damaged mitochondria and invasive microorganisms are ubiquitinated, and SQSTM1 is phosphorylated at Ser407 and Ser403 sequentially. To deliver its cargo for autophagic degradation, SQSTM1 binds to the autophagosome-localized protein LC3, which plays multiple roles in autophagy, including membrane fusion, cargo selection and autophagosome transport (Katsuragi et al., 2015; Yamada et al., 2019; Aparicio et al., 2020). The LIR motif within NDP52 is dispensable for ATG8 recruitment and specificity during PINK1/Parkin mitophagy, and the additional recruitment of NDP52 amplifies mitophagy through an ATG8-dependent positive feedback loop (Padman et al., 2019). Ectopic placement of NDP52 on mitochondria is sufficient to initiate mitophagy by focally localizing and activating the ULK1 (unc-51 like autophagy activating kinase) complex. The ability of NDP52 to induce mitophagy depends on its interaction with the ULK1 complex, which is facilitated by TBK1 as the primary driver of targeted autophagy autophagosome biogenesis (Vargas et al., 2019). Mitochondrial profusion protein Mitofusins (MFN1 and MFN2), which were found to be a target for Parkin mediated ubiquitination, are transmembrane GTPase embedded in the outer membrane of mitochondria (Basso et al., 2018). Parkin can mediate ubiquitination and proteasomal degradation of MFN1 and MFN2, but mitophagy can also be triggered by Parkin in MFN1/MFN2 double knockout cells, suggesting that Mitofusin ubiquitination and proteasomal degradation are not essential to mitochondrial activation. MFN1 seems to be more rapidly degraded than MFN2 via Parkin, and this may be related to the differential activity of the two proteins in mitochondrial fusion (Tanaka et al., 2010; Song et al., 2015). Autophagy of NDP52 and TAX1BP1 is adjusted by TBK1, to which the kinase may bind through the articulatory NAP1 (nucleosome assembly protein 1) (Fu et al., 2018). NAP1 involves binding to the SKICH (SKIP carboxyl homology)-containing autophagy receptor TAX1BP1 (Thurston et al., 2009).

**TABLE 1:** Brief description of mitophagy receptors.

Locations	Receptors	Function	References
OMM	OPTN	Forming a complex with ATG9A vesicles	Heo et al., 2015; Yamano et al., 2020
OMM	SQSTM1/P62		Yamada et al., 2019
OMM	CALCOCO2/NDP52	Amplifying mitophagy through an Atg8-dependent positive feedback loop	Goiran et al., 2018; Padman et al., 2019
OMM	MFN1/2		Chen and Dorn, 2013; Song et al., 2015
OMM	TAX1BP1		Heo et al., 2019
OMM	BNIP3L/NIX	Owning the unique ability to interact with processed MAP1LC3B	Novak et al., 2010; Hanna et al., 2012; Liu et al., 2012; Springer and Macleod, 2016
OMM	FUNDC1		
OMM	BNIP3		
OMM	VDAC	Mediating degradation of mitochondria in PINK1- and PRKN-dependent signaling pathway	Chen and Dorn, 2013
OMM	RHOT1		
IMM	Cardiolipin	Mediating ubiquitin independent receptor-mediated mitophagy	Cho et al., 2020
IMM	PHB2		

Other mitophagy receptor proteins, such as BNIP3L/NIX (BCL2 interacting protein 3 like), FUNDC1 (FUN14 domain containing 1), and BNIP3 (BCL2 interacting protein 3), localized on the mitochondrial outer membrane and, thus, own the unique ability to interact with processed LC3 independent of ubiquitin (Novak et al., 2010; Hanna et al., 2012; Liu et al., 2012; Springer and Macleod, 2016). BNIP3L, a BH3-only proapoptotic protein beneficial to ischemic brain injury, is indispensable for mitochondrial clearance during reticulocyte maturation and is also involved in mitophagy under hypoxia in a variety of cells (Xiang et al., 2017; Yuan et al., 2017). DNM1L (dynamin 1 like) is a cytoplasmic molecule that is recruited to mitochondria to orchestrate mitochondrial fission or fusion and mitophagy (Vásquez-Trincado et al., 2016; Liu et al., 2020). PGAM5 (PGAM family member 5) dephosphorylates FUNDC1 at serine 13 to enhance FUNDC1 interaction with LC3, whereas CK2 (creatine kinase 2) phosphorylates FUNDC1 to reverse the effect of PGAM5 (Chen et al., 2014; Chen et al., 2016). BNIP3, a BCL2 family protein with an atypical BH3 domain, plays an important role in the interaction of BNIP3 with BCL2 (BCL2 apoptosis regulator), which plays a pro-survival role under certain pathological conditions (Zhang and Ney, 2009; Tang C. et al., 2019). In addition, TBK1 has recently been found to phosphorylate autophagy receptors, thereby producing signal amplification during mitophagy (Richter et al., 2016). Overall, mitophagy plays a beneficial protective role in the quality control of mitochondria not only by autophagic receptors but also through mitochondrial dynamics to maintain human health.

## Mitophagy in Sepsis

Sepsis is a systemic inflammatory response syndrome caused by infection, associated with acute organ dysfunction and a high risk of death (Cecconi et al., 2018). Organ failure and increased mortality are most likely related to the metabolic, immunological, and autonomic features of sepsis. However, it is an oversimplification to attribute these to single inflammatory pathways. No positive result was obtained in clinical trials regarding TNF-α (anti-tumor necrosis factor-α) antibodies, high-dose steroids, and activated protein C (Nunnally, 2016). There is growing evidence that autophagy is associated with the elimination of invading pathogens and the maintenance of a stable inflammatory response following the induction of multiple pathogens or their associated products, such as viral DNA or LPS (lipopolysaccharide). PRRs (Pattern recognition receptors) sense exogenous threats or endogenous stress, recent studies have demonstrated a link between PRRs and autophagy (Oh and Lee, 2014). Xu et al. (2007) found that stimulation of TLR4 with LPS induces autophagosome formation via the TRIF–p38 axis whereas lipoprotein acid binding to TLR2 induces autophagy through the MAPK1/ERK2-MAPK3/ERK1 pathway. Autophagy is increased in the early stages of sepsis, but autophagic flux decreases in the later stages, which promotes organ damage (Pua et al., 2007; Chien et al., 2011; Hsieh et al., 2011). Impaired autophagy confirmed by silencing ATG7 with siRNA exacerbates TNF (tumor necrosis factor)-induced DNA fragmentation in proximal renal tubular cells and hepatocytes (Pua et al., 2007; Chien et al., 2011). This implies that autophagy is an extremely valuable therapeutic target in sepsis. Insufficient autophagy does lead to uncontrolled infection and excessive inflammation by enhancing caspase-1 activation and increasing IL-1β production and secretion, both of which are major causes of sepsis (Zhong et al., 2016). Notably, one of the most important issues in mitophagy therapy strategies is the proper timing, we suggest that LC3 II and p62 can be used to monitor autophagic flux in septic patients, which are significant markers acknowledged by many studies (Ho et al., 2016; Yin et al., 2017). However, many studies have shown that autophagy plays a different role in organ protection in sepsis, and autophagy may have an opposite role in skeletal muscle protection (Yin et al., 2019). During sepsis, amino acid supplementation antagonizes the activation of skeletal muscle autophagic signaling and prevents sepsis-induced muscle protein degradation (Hernandez-García et al., 2016).

Mitochondria are more than a simple powerhouse of cells. Mitochondria play a key role in Ca^2+^ homeostasis, triggering the apoptosis/necrosis pathway and generating ROS to regulate cell fate. In addition, mitochondrial ROS and mtDNA can activate NLRP3 inflammasome, which links mitochondria to sepsis (García et al., 2015; Acuña-Castroviejo et al., 2017). Multiple studies have demonstrated that sepsis-induced mitochondrial alterations may play a pathophysiological role in the induction and propagation of sepsis-induced organ failure (Singer, 2007; Exline and Crouser, 2008; Duran-Bedolla et al., 2014; Thiessen et al., 2017; Lelubre and Vincent, 2018). So, mitophagy has a significant effect on sepsis with eliminating dysfunctional mitochondria. For instance, in a mouse model of *Staphylococcus aureus*-induced pneumonia, mitophagy are extensively activated in the alveolar region, and the mitochondrial quality control processes promote the ability of lung cells to eliminate and replace damaged mitochondria and thereby support cell survival (Suliman et al., 2017). Mitochondria are susceptible to damage in sepsis, and the mitochondrial inner membrane potential decreases (Zhang et al., 2018). Damaged mitochondria are separated by autophagosomes and eventually degraded by fusion with lysosomes, thereby facilitating the recovery of septic organ function (Pan et al., 2018). SESN2 (sestrin2), called stress-inducible protein, suppresses prolonged NLRP3 inflammasome activation in macrophages by increasing ULK1 protein levels to activate mitophagy and thereby clear damaged mitochondria. SESN2 knockout mice exhibited impaired mitophagy and septic mice exhibited excessive activation of the inflammatory body and increased mortality (Kim et al., 2016). In addition, restricting inflammasome activation in macrophages by increasing mitophagy and decreasing mitochondrial ROS might be a crucial mechanism for MSCs (mesenchymal stromal cells) to defend against sepsis (Li et al., 2018). In critically ill patients, Patoli et al. found that blood monocytes from septic patients had inhibited mitophagy compared to those from non-septic patients. This work suggested that mitophagy inhibited myeloid cell activation and worsen sepsis outcome (Patoli et al., 2020). Mitophagy is critical in combating oxidative stress during the development of sepsis, and it is one of the most studied types of selective autophagy of organelles. Accumulating evidences suggest that mitophagy may become a new potential target for sepsis treatment.

## Mitophagy Is Able to Mitigate Organ Dysfunction in Sepsis

The pathogenesis of sepsis is extremely complex, with mechanisms at the cellular and molecular level such as mitochondrial damage, imbalance in the inflammatory response, abnormal immune function, abnormal neuroendocrine immune networks, endoplasmic reticulum stress, autophagy and other pathophysiological processes that ultimately result in organ dysfunction (Table 2), such as heart, kidney, lung and liver (Lelubre and Vincent, 2018; Huang et al., 2019). Recent studies have implied that mitophagy may be activated to protect against infection and organ dysfunction (Figure 2). However, there is an experiment demonstrate that inhibition of mitophagy drives macrophage activation and may enhance host defense and reverse sepsis-induced immunoparalysis (Patoli et al., 2020).

**TABLE 2:** The protective effects of mitophagy on different organs of sepsis.

Organ	Organelle dysfunction	Protective effects	References
Heart	Dysfunction of mitochondria	Controlling over inflammation by reducing mitochondrial DAMPs to improve whole-organ activity in the heart Improving myocardial function via promoting mitochondrial biogenesis	Oka et al., 2012; Laker et al., 2017
Kidney	Dysfunction of mitochondria	Promoting a decrease in the levels of NLRP3 and the caspase cascade to protect against renal injury Reducing renal ischemic injury and restoring tubular reabsorption	Tang C. et al., 2019; Xu et al., 2019
Lung	Dysfunction of mitochondria	Removing excess ROS to recover mitochondrial oxidative phosphorylation to provide energy for lung Attenuating excessive inflammatory response of small airway epithelial cells	Singer, 2014
Liver	Dysfunction of mitochondria	Degrading damaged mitochondria and preventing apoptosis to improve liver function	Carchman et al., 2013
			

**FIGURE 2:** Mitophagy in sepsis-induced organ injury. **(A)** Beclin-1 contributes to the inhibition of BNIP3L- and BNIP3- mediated mitophagy, while promoting PINK1-Parkin dependent mitophagy, which can reduce mitochondrial DAMPs and control inflammation to improve septic cardiac dysfunction. TSG101 can also prevent myocardial injury by promoting Parkin-induced mitophagy. **(B)** BNIP3 overexpression has been shown to induce mitophagy and TRPA1 regulates mitochondrial biogenesis and mitophagy. OPTN is an important articulator of the PINK1-PARK2 pathway of mitophagy in septic AKI. These molecules all reduce NLRP3 inflammasome activation and apoptosis to prevent sepsis-induced kidney injury. **(C)** MKK3 deficiency appears to increase mitophagy through PINK-1-Parkin pathway. Both BCL2 overexpression and Bad knockdown alleviate septic lung injury and inhibit mitophagy, with improving survival. **(D)** Rg3 regulates mitophagy which ameliorates mitochondrial dysfunction and protects against sepsis-induced liver damage. HO-1 enhances Parkin- and BNIP3-mediated mitophagy and H_2_ gas promotes mitophagy through FUNDC1-dependent manner to attenuate septic liver injury.

### Mitophagy Can Improve Cardiac Dysfunction by Reducing Mitochondrial DAMPs in Sepsis

Cardiac dysfunction is an established and severe component of multi-organ failure associated with sepsis. Recent studies suggest that damage to autophagy and organelle-specific autophagy may account for contractile dysfunction and apoptotic cell death in cardiomyocytes. Mitophagy presents a control over inflammation by reducing mitochondrial DAMPs (danger-associated molecular patterns) (Oka et al., 2012). The impact of mitochondria and mitophagy on the regulation of inflammation has received widespread attention in recent years. Mitochondria are major participants in innate immunity, and cytoplasmic mtDNA fragments stimulate the DNA sensor cGAS and promote the STING-IRF3-dependent pathway, thereby enhancing type I interferon responses and conferring broad viral resistance (West et al., 2015). The synthesis of mtDNA, induced after the engagement of Toll-like receptors, is essential for NLRP3 signaling, and cytoplasmic oxidized mtDNA is associated with the NLRP3 inflammatory vesicle complex and is required for its activation (Zhong et al., 2018). Therefore, mitophagy is expected to be an effective approach to reduce mitochondrial DAMPs and control inflammation to improve septic outcome.

Hsieh et al. (2011) concluded there was increased formation of autophagosomes whereas decreased degradation of autophagosomes in the left ventricle 24 h after cecal ligation and puncture (CLP) (Baker et al., 1983), indicating incompletion of the autophagic process. Notably, rapamycin can lead to the completion of the autophagic process, which may play a cardioprotective role in sepsis (Hsieh et al., 2011). However, it has also been suggested that the inhibition of autophagy contributes to the recovery of myocardial contractile function (Pang et al., 2019). This provides valuable ideas and new insights for addressing cardiac dysfunction in sepsis. The content of mitochondria is high in the myocardium and can provide sufficient energy for myocardial activity. Impaired mitochondrial structure and function, associated with the overproduction of mitochondrial mtROS and the production of mitochondria-derived DAMPs, play a key role in the induction of cardiac inflammation and functional defects during sepsis (Zang et al., 2007, 2012a). Zang et al. (2012b) indicated that targeted removal of mtROS protects mitochondrial function, reduces inflammation and improves whole-organ activity in the heart during sepsis. Beclin-1, one of the first identified mammalian autophagic effectors, is a central player in autophagy and constitutes a molecular platform that regulates autophagosome formation and maturation (Liang et al., 1999; Hill et al., 2019). Fernández et al. (2018) suggested that activation of the beclin-1 class III PI3K autophagy-initiating complex may be an efficient and secure way to bypass upstream senescence signaling, which can extremely promote mammalian health and lifespan. In particular, disruption of Beclin-1-BCL2 binding may have substantial beneficial effects on mammalian lifespan and healthspan (Fernández et al., 2018). Beclin-1 levels affect the autophagic response to sepsis and mTOR signaling in the heart. In addition, Beclin-1 may contribute to the inhibition of receptor-mediated (such as BNIP3L and BNIP3) activation of mitophagy, while increasing LC3II associated with the mitochondrial and PINK1-Parkin pathways by promoting a more adaptive mitochondrial response via PINK1/Parkin (Sun et al., 2018). In addition to activating mitophagy to remove damaged mitochondria, beclin-1 may promote mitochondrial biogenesis through upregulation of PINK1/Parkin and/or AMPK/ULK1 (Ivankovic et al., 2016; Laker et al., 2017; Marin et al., 2017) and improve myocardial function. Knockdown of Beclin-1 attenuates the beneficial effects of CO on reducing inflammation and decreasing bacteremia. Therefore, the protective effect of Beclin-1 during sepsis does not seem to be limited to the heart. Significantly, park2 is an important player in mitophagy, and park2 deficiency is associated with mild mitochondrial dysfunction and, more importantly, impaired recovery from sepsis-induced mitochondrial and cardiac dysfunction (Piquereau et al., 2013). In addition, TSG101 (tumor susceptibility gene 101) is a crucial member of the endosomal recycling complex required for transport, which may affect autophagic flux. It has been recently shown that elevated TSG101 can prevent endotoxin-triggered myocardial injury by promoting Parkin-induced mitophagy (Anding et al., 2018; Essandoh et al., 2019), which has the potential to be a new target for the treatment of myocardial dysfunction in sepsis.

Dysfunction of other organelles, such as ER (endoplasmic reticulum), also contributes to the abnormal phenotype of cardiomyocytes and is one of the important factors in septic inflammation. As with mitochondrial dysfunction, ER stress contributes to poor myocardial performance by promoting the development of inflammation in sepsis (Zhang J. et al., 2020). Thus, reducing ER stress can improve cardiomyocyte viability. Administration of the ER stress inhibitor 2-aminopurine improves cardiac pathology, suggesting that maintaining functional homeostasis of the ER may be a priority for cardiomyocyte viability and response (Ayyappan et al., 2019). However, the implication of reticulophagy in septic heart disease are still utmostly unclear.

### Mitophagy Was Enhanced in the Earlier Stage of Sepsis to Protect Against Kidney Injury

Kidney is one of the most common organs injured in sepsis, leading to sepsis-associated acute kidney injury (SA-AKI), which increases the morbidity and mortality of sepsis. Furthermore, patients with AKI associated with sepsis had a significantly increased mortality rate compared to patients with AKI of other etiologies (Poston and Koyner, 2019). Sunahara et al. (2018) confirmed that in CLP-induced acute kidney injury, the LC3-II/LC3-I ratio increased at 6–8 h, while the number of LC3-II/LC3-I significantly decreased at 24 h (Sunahara et al., 2018). Rapamycin induced autophagy and may reduce AKI in sepsis. Autophagy plays various roles in the inflammatory response and has great potential to protect kidney from multiple kidney inflammatory insults (Kimura et al., 2017).

Recently, the significance of selective autophagy has been emphasized in disease processes, as the targets of selective autophagy include key organelles associated with disease, such as mitochondria. Remarkably, disrupted renal bioenergetics plays a key role in the AKI process of CLP mice (Yang et al., 2014), which is closely related to the activity of mitochondria. Because in the process of reabsorption and secretion of anti-chemical gradient, renal tubule cells need a large number of mitochondria to supply ATP, which leads to mitochondria disorder and damage under stress conditions (Liu et al., 2019). Mitophagy was enhanced in the earlier stage of AKI in sepsis, characterized by elevated levels of LC3 and increased co-localization of COXIV and LC3. However, this protective effect was compromised at a later stage and was accompanied by reduced Pink1 and Parkin levels, and the co-localization of COXIV and LC3 decreased (Liu et al., 2019). The fusion of functionally impaired mitochondrial was suppressed, while fission was increased in AKI, which can be ameliorated by OPA1 overexpression or Drp1 blockade (Perdiz et al., 2017; Garcia et al., 2018). Mitochondrial division inhibitor-1 (Mdivi-1), a pharmacologic inhibitor of Drp1, can block subsequent AKI progression (Sun et al., 2019). It has been demonstrated that activation of mitophagy promotes a decrease in the levels of NLRP3 and the caspase cascade (Xu et al., 2019), while activation of NLRP3 and proteins of the caspase family, such as caspase-1 and caspase-3, inhibit mitophagy and therefore exacerbate inflammation and cellular damage. A recent study noted that TRPA1 (transient receptor potential anchor protein 1) prevents sepsis-induced kidney injury by regulating mitochondrial biogenesis and mitophagy (Zhu et al., 2018). Mitophagy mediated by the mitochondrial receptor BNIP3 has also been shown in renal tubular cells with ischemic AKI (Tang C. et al., 2019). Of interest, BNIP3 overexpression has been shown to induce mitophagy, suggesting that mitophagy can be mediated through the HIF-1/BNIP3 pathway in renal tubular cells during AKI (Parikh et al., 2015). Sepsis caused more serious kidney injury and apoptosis in pink1 or park2 knockout mice than in wild-type mice, suggesting a beneficial role for mitophagy in septic AKI. Furthermore, knockdown of OPTN diminishes mitophagy, suggesting that OPTN is an important articulator of the PINK1-PARK2 pathway of mitophagy in septic AKI, which provides new insights into the molecular pathway of mitophagy in septic AKI (Wang et al., 2021). Although no clear mechanism of mitophagy has been identified in septic AKI, we believe that mitophagy could be a promising therapeutic target in septic AKI and should be taken into consideration for further researches.

### Increased Mitophagy Contribute to Alleviated Lung Injury via Eliminating Excessive ROS in Sepsis

Among the organs impaired in sepsis, the lung is the first and most common organ to be injured. Concomitant ARDS (acute respiratory distress syndrome) is one of the most critical prognostic factors for death in patients with sepsis. The clinical outcome of sepsis-associated ARDS is worse than that of non-sepsis-associated ARDS (Park et al., 2019). It is widely believed that inflammation and apoptosis of lung epithelial cells play a crucial role in the pathogenesis of ARDS, and it has been reported that LPS-induced apoptosis can be counteracted by rapamycin-induced cellular autophagy (Ji et al., 2018). Another study found that AMPK activator might activate mitochondrial biogenesis by increasing PGC-1α expression, thereby promoting lung recovery. AMPK activator treatment further increased the expression of autophagy-related proteins, suggesting that increased autophagy may be an additional protective mechanism to attenuate sepsis-induced lung injury (Kitzmiller et al., 2019). Increased mitophagy may also play a role in lung protection. Nrf2 protein levels were significantly increased and alveolar mitophagy was activated 6 h after CLP in mice (Yin et al., 2019). In addition, the protective effect of GAPDH (glyceraldehyde-3-phosphate dehydrogenase) against sepsis-associated lung injury is mediated by enhanced ATG12-dependent autophagy (Colell et al., 2007; Takaoka et al., 2014).

More specifically, not only autophagy, but mitophagy also has important implications for ARDS. ARDS is accompanied by a severe inflammatory response and is associated with oxidative stress caused by excessive ROS production (Galley, 2011). Uncontrolled generation of ROS eventually overwhelms the cell and causes morphological damage, especially to the mitochondria. More specifically, this excessive ROS production directly inhibits mitochondrial oxidative phosphorylation (Singer, 2014). Inflammation leads to excessive ROS production and damage to mitochondria, which will lead to apoptosis of lung epithelial cells, epithelial barrier destruction and the development of ARDS. Nrf2 (Nuclear factor E2-related factor 2) is responsible for mitochondrial quality control via defensing against oxidative stress in lung (Chang et al., 2015). Nrf2 knockdown produces reduced LC3-II and selective autophagy receptor protein p62, suggesting a key role for Nrf2 in redox-sensitive mitophagy. Furthermore, mitophagy in the alveolar region appears to rely on the activation of Nrf2 (Chang et al., 2015). Therefore, we believe that Nrf2 may be an effective treatment for ARDS in sepsis. In addition, MKK3 deficiency appears to increase both mitochondrial biogenesis and mitophagy through the action of Sirt1, Pink1 and Parkin. This leads to a more robust mitochondrial network that provides protection against septic ARDS (Mannam et al., 2014). Zhang et al. demonstrated that BCL2 protein regulates mitophagy in LPS-induced ARDS by modulating the PINK1/Parkin signaling pathway in 2020. Both BCL2 overexpression and Bad knockdown were reported to inhibit apoptosis and mitophagy, alleviate LPS-induced lung injury and improve survival (Zhang Z. et al., 2020). Although there are few studies on mitophagy in sepsis-associated lung injury, we believe this will provide new insights in investigating treatment strategies for sepsis-associated lung injury.

### Increased Mitophagy in Liver Can Control Mitochondrial Mass to Improve Liver Function in Sepsis

The liver plays a crucial role in sepsis because it has vital metabolic functions. It is also essential in immune defense, and usually acts as a target of dysregulated inflammation (Protzer et al., 2012). The liver represents a key element of the anti-microbial response and dysregulation of this complex interface leads to sepsis-induced liver injury and increased sepsis-related mortality (Strnad et al., 2017). It has been well accepted that autophagy is an important protective mechanism in septic liver injury. The increased autophagic response against LPS in hepatocytes depends on the MAPK/p38 and BECN1 complex signaling, but not on the classical autophagic signaling (MTOR-ULK1). Inhibition of LPS-induced autophagy increased hepatic lipid accumulation and inflammation in mice (Chung et al., 2017), suggesting that autophagy contributes to the maintenance of homeostasis of lipid metabolism and protection of liver function during sepsis. Cho et al. (2016) suggested that genipin restores impaired autophagic flux to protect against septic liver injury via attenuating the levels of calpain 1 and cleaved Atg5, but not mTOR. In addition, circulating (carbomyl phosphate synthase)-1 is a marker of hepatic mitochondrial damage and depletion in the subacute phase of CLP sepsis. Mitochondrial depletion is not caused by cell death but is apparently associated with autophagic clearance of damaged mitochondria (Crouser et al., 2006). Strong evidences demonstrated that autophagy occurs in the liver during the first 4 h after CLP, but decreases thereafter until 24 h (Ho et al., 2016).

Mitophagy has also been reported to be involved in the pathogenesis of septic liver injury. It has been experimentally confirmed that hepatocyte mitochondrial density is reduced after LPS treatment. Mitophagy is increased in the liver in sepsis to control mitochondrial mass to improve liver function (Carchman et al., 2013). Another study also found that increased mitophagy in sepsis has a protective effect on liver function. Ginsenoside Rg3 regulates mitophagy by activating the AMPK signaling pathway, thereby ameliorating mitochondrial dysfunction and protecting against sepsis-induced cell and organ damage. Mitochondrial protective function was reduced in LPS-induced human primary hepatocyte injury after treatment with autophagy inhibitors or AMPK inhibitors (Xing et al., 2017). Heme oxygenase (HO)-1 is a cytoprotective enzyme that is upregulated under cellular stress and its expression was increased in whole liver and mitochondria during sepsis. HO-1 enhances Parkin- and BNIP3-mediated mitophagy to attenuate septic liver injury by regulating TLR4-mediated mitochondrial QC during sepsis (Park et al., 2018). Interestingly, molecular hydrogen (H_2_) plays a beneficial role as an antioxidant in sepsis. A study reported that the inhalation of H_2_ gas promoted mitophagy through the regulation of FUNDC1-dependent manner and protected mice from the sepsis-induced liver injury. The protective effect of H_2_ on liver injury in sepsis could be effectively reversed by the FUNDC1 inhibitor (Yan et al., 2019).

## Conclusion and Clinical Perspectives

Autophagy, a conserved catabolic process, is one of the innate immune defense mechanisms against microbial challenges. As the center of energy metabolism, mitochondria have a major role in maintaining homeostasis and triggering apoptosis. However, damaged mitochondria can produce excessive ROS to jeopardize cells, which will be scavenged by mitophagy via PINK1-Parkin-dependent and -independent pathways. Mitophagy indicates immensely significant benefits in the defense against infection through the quality control of specific organelles, thereby maintaining the survival and function of cells. Sepsis causes multiple organ dysfunction in its most severe form that can generate a state of chronic critical illness. It seems an apocalyptic day for the human bodies without effective treatment. Mitochondria are susceptible to damage in sepsis, and there may be a significant relationship between damaged mitochondria and the pathophysiology of septic organ failure. Mitophagy can selectively eliminate “innocent bystanders” to ensure the normal function of organs during sepsis, and thereby provide a new therapeutic target for sepsis induced organ dysfunction.

It is noteworthy that the interplay between multiple organelles is also critically involved in sepsis. Dysfunction of mitochondria is noted in a septic animal model, which presents with evident derangement of ER and intractable ER stress. UCP2 (Uncoupling protein 2), an important mediator of the transportation of calcium, has been shown to transfer calcium from the ER to mitochondria (Dromparis et al., 2013). Moreover, the expression of UCP2 has been a promising therapeutic target for sepsis due to its great capacity in regulating NLRP3 inflammasome (Moon et al., 2015), and the targeted induction of UCP2-mediated autophagy may also have important therapeutic potential (Tang R. et al., 2019). What is the situation of mitochondria and ER in septic organ dysfunction and whether there is a collaborative relationship between two specific autophagy, mitophagy, and reticulophagy, which we do not clearly understand yet. These questions should be further elucidated in terms of specific autophagy and clinically relevant significance, as it may be a potential therapeutic target for septic organ dysfunction.

## Author Contributions

C-lZ, R-qY, and L-xL conducted the literature review and drafted the manuscript, which J-fW and X-mD conceptualized, supervised, and revised. All the authors read approved the final manuscript.

## Conflict of Interest

The authors declare that the research was conducted in the absence of any commercial or financial relationships that could be construed as a potential conflict of interest.

## Abbreviations

ARDS: acute respiratory distress syndrome
ATG: autophagy related
ATM: ataxia-telangiectasia-mutated
BCL2: BCL2 apoptosis regulator
BNIP3: BCL2 interacting protein 3
BNIP3L/NIX: BCL2 interacting protein 3 like
CALCOCO2/NDP52: calcium binding and coiled-coil domain 2
CLP: cecal ligation and puncture
DAMPs: danger-associated molecular patterns
ER: endoplasmic reticulum
FUNDC1: FUN14 domain containing 1
IMM: inner mitochondrial membrane
MAP1LC3/LC3: microtubule associated protein 1 light chain 3
MFN1: mitofusin 1
MFN2: mitofusin 2
NLRP3: NLR family pyrin domain containing 3
Nrf2: Nuclear factor E2-related factor 2
OMM: outer mitochondrial membrane
OPTN: optineurin
PINK1: PTEN induced putative kinase 1
PGAM5: PGAM family member 5
PRKN: Parkin RBR E3 ubiquitin protein ligase
RBR: RING-in-between-RING
ROS: reactive oxygen species
SESN2: sestrin2
SQSTM1/p62: sequestosome 1
TAX1BP1: Tax1 binding protein 1
TBK1: TANK binding kinase 1
TUFm: mitochondrial Tu translation elongation factor
UCP2: Uncoupling protein 2
ULK1: unc-51 like autophagy activating kinase.
